RETRACTED

# New insights into molecular signaling pathways and current advancements in prostate cancer diagnostics & therapeutics

**DOI:** 10.3389/fonc.2023.1193736

**Published:** 2023-08-17

**Authors:** Neha Thakur, Sameer Quazi, Bindu Naik, Saurabh Kumar Jha, Pallavi Singh

**Affiliations:** ^1^ Department of Biotechnology, Graphic Era (Deemed to be University), Dehradun, Uttarakhand, India; ^2^ Department of Chemistry, Akshara First Grade College, Bengaluru, India; ^3^ GenLab Biosolutions Private Limited, Bangalore, Karnataka, India; ^4^ Department of Biomedical Sciences, School of Life Sciences, Anglia Ruskin University, Cambridge, United Kingdom; ^5^ School of Health Sciences, Faculty of Biology, Medicine and Health, The University of Manchester, Manchester, United Kingdom; ^6^ Solution Chemistry of Advanced Materials and Technologies (SCAMT) Institute, ITMO University, St. Petersburg, Russia; ^7^ Department of Food Science and Technology, Graphic Era Deemed to be University, Dehradun, Uttarakhand, India; ^8^ Department of Biotechnology, School of Engineering and Technology, Sharda University, Greater Noida, India; ^9^ Department of Biotechnology Engineering and Food Technology, Chandigarh University, Mohali, India; ^10^ Department of Biotechnology, School of Applied & Life Sciences (SALS), Uttaranchal University, Dehradun, India

**Keywords:** prostate cancer, androgen deprivation therapy, castration resistant prostate cancer, RISUG adv, poly ADP ribose polymerase, AR signaling, PI3K

## Abstract

Prostate adenocarcinoma accounts for more than 20% of deaths among males due to cancer. It is the fifth-leading cancer diagnosed in males across the globe. The mortality rate is quite high due to prostate cancer. Despite the fact that advancements in diagnostics and therapeutics have been made, there is a lack of effective drugs. Metabolic pathways are altered due to the triggering of androgen receptor (AR) signaling pathways, and elevated levels of dihydrotestosterone are produced due to defects in AR signaling that accelerate the growth of prostate cancer cells. Further, PI3K/AKT/mTOR pathways interact with AR signaling pathway and act as precursors to promote prostate cancer. Prostate cancer therapy has been classified into luminal A, luminal B, and basal subtypes. Therapeutic drugs inhibiting dihydrotestosterone and PI3K have shown to give promising results to combat prostate cancer. Many second-generation Androgen receptor signaling antagonists are given either as single agent or with the combination of other drugs. In order to develop a cure for metastasized prostate cancer cells, Androgen deprivation therapy (ADT) is applied by using surgical or chemical methods. In many cases, Prostatectomy or local radiotherapy are used to control metastasized prostate cancer. However, it has been observed that after 1.5 years to 2 years of Prostatectomy or castration, there is reoccurrence of prostate cancer and high incidence of castration resistant prostate cancer is seen in population undergone ADT. It has been observed that Androgen derivation therapy combined with drugs like abiraterone acetate or docetaxel improve overall survival rate in metastatic hormone sensitive prostate cancer (mHSPC) patients. Scientific investigations have revealed that drugs inhibiting poly ADP Ribose polymerase (PARP) are showing promising results in clinical trials in the prostate cancer population with mCRPC and DNA repair abnormalities. Recently, RISUG adv (reversible inhibition of sperm under guidance) has shown significant results against prostate cancer cell lines and MTT assay has validated substantial effects of this drug against PC3 cell lines. Current review paper highlights the advancements in prostate cancer therapeutics and new drug molecules against prostate cancer. It will provide detailed insights on the signaling pathways which need to be targeted to combat metastasized prostate cancer and castration resistant prostate cancer.

RETRACTED

## 1 Introduction

The lack of precise therapeutics for cancer still haunts us in the age of advanced medical therapeutics, when the scientific community has discovered the cure for the most fatal diseases affecting human lives. Leading the source for the development of cancer are the unregulated molecular signaling pathways and the disruption of metabolic machinery, which hamper the normal growth of the cells. Despite medications, chemotherapy, and operative procedures, carcinoma cells re-establish themselves within the body within a certain period of time (1). Prostate adenocarcinoma accounts for more than 20% of deaths related to cancer in males, and it is the fifth-leading cancer diagnosed in males across the globe (2, 3). Despite every advancement in therapeutics and diagnostics, effective drugs against cancer cells are still not available on the global market (4). Metabolic pathways are altered due to the triggering of androgen receptor signaling pathways. AR is a transcription factor that responds to ligands, and the presence of AR splice variants introduced another degree of complexity, with some showing constitutive activity as well as ligand-independent activity (5). Almost every case, or approximately 90% of cases, shows a confined organ, and it may change location in the specific organ during diagnosis. The prostate-specific antigen (PSA) and clinical stages are the parameters on which decisions will be made to go for regular surveillance of the patient, prostatectomy, or local radiotherapy (**Figure 1**) (6). Androgen deprivation therapy via chemical castration or surgical means is done if the cancer has spread beyond the boundaries of the prostate, just to ensure the decrement in circulatory levels of testosterone (7). ADT’s effects are very temporary, and most patients will acquire resistance within 18 to 36 months after starting treatment, eventually progressing to castration-resistant prostate cancer (8). With the use of cognate ligand dihydrotestosterone (DHT) competitive antagonists, AR function is blocked directly so as to achieve deprivation of androgen at the maximal range, whereas in the CRPC and the therapeutic course of action, AR axis is an essential part (9, 10). At present, studies are done clinically with different second-generation antagonists of AR, which are given in combination with another drug or as a single agent (11). Recently, it has been approved that sipuleucel-T, an immunotherapy that is cell-based, and taxanes be used as additional therapies for metastatic CRPC (mCRPC). Radium-223 dichloride is used with targeted alpha therapy for mCRPC treatment, and it’s beneficial for the treatment (12). Thereafter, several advancements occur before the relapse of disease occurs, in which the mechanisms of resistance, including all the causes that can successfully block AR signaling, include: - gene amplification of AR; - AR cofactors with altered levels; - androgen levels increasing locally; - variants, splice sites, and LBD mutations (13). Multiple pathways are associated with prostate cancer, as survival pathways and growth-promoting pathways interact with AR signaling. Many scientific investigations have prominently demonstrated the roles of the Ak-strain transforming (AKT) pathway, the phosphoinositide 3-kinase (PI3K), an enzyme, and a mechanistic target of rapamycin (mTOR), the pathway, in the repair of damaged DNA (14). Clinical studies have revealed that AR signaling, when intermingled with a compound, results in a combination that approaches specific inhibitors with a single agent (15). In prostate cancer, a large number of epigenetic markers such as DNA methylation, acetylation, and histone methylation have been reported (16). The compounds that communicate with epigenetic targets include bromo- and extra-terminal (BET) proteins or the polycomb repressive complex 2 (PRC2) proteins, and currently, these molecules have entered clinical trials. Researchers are evaluating immune checkpoint inhibitors in CRPC due to the astounding success of immunotherapies in treating cell and melanoma lung cancer (17). Hereditary factors contribute to enhanced risks of acquiring prostate cancer from one generation to the next (18). The medication and treatments are more precise in determining the most accurate therapeutics for a particular cancer patient (19). The collaborative endeavors by various government agencies, genome scientists, and pharmaceutical companies will definitely provide a promising cure and better medications for prostate cancer treatment. Also, the CRPC is a lethal disease (20). It mainly occurs in the metastatic or advanced disease of patients with prostate cancer (21). While facing all the challenges of the search for therapeutics, a compound named RISUG, a polymeric male contraceptive, was noted to have an anti-cancerous effect based on its chemical and physical properties. Singroul et al. (2020) observed the minimum incubation time required for 10 mg/ml RISUG in DMSO to demonstrate the anti-cancer effect on PC3 prostate cancer cells evaluated via MTT assay for the duration of 72h (22). The current review focuses on advancements in prostate cancer therapeutics as well as the molecular signaling pathways involved in boosting the occurrence of prostate cancer.

RETRACTED

**Figure 1:** Visualization of stages involved in human prostate cancer.

## 2 Tumor microenvironment: the cross-talk between PC cells and carcinoma-associated fibroblasts and macrophages

Fibroblasts represent the predominant cellular constituents of the connective tissue. During the process of wound healing, fibroblasts undergo a phenotypic transformation into an activated state. Activated fibroblasts exhibit specific features that are reminiscent of both fibroblasts and smooth muscle cells. Tumors are frequently comparable to non-healing wounds in numerous instances (23). The regenerative mechanism of stromal cells initiated by cancer cells exhibits certain resemblances with the process of wound healing. Cancer is characterized by the presence of activated fibroblasts, which are referred to as cancer-associated fibroblasts (CAFs). CAFs are not the same as regular fibroblasts, which have specific markers, heightened pro-tumorigenic qualities, and the ability to create a wide range of pro-inflammatory substances. CAFs even have the ability to attract different kinds of stromal cells to the main lesion as well as metastatic lesions that are caused by cancer. They all have a role in the formation of the cancer microenvironment, which helps to promote the growth of tumors, as well as their invasion and dissemination. The precise origin of CAFs as well as the methods by which normal cells transform into CAFs are not yet fully understood; nonetheless, the available information suggests that a sizeable portion of CAFs are derived from normal fibroblasts that are located in close proximity to cancer cells and are in constant interaction with these cells. Multiple signal axes seemed to be abnormally active in CAFs in comparison to normal fibroblasts. The possibility that primary grown CAFs may maintain their phenotypic over the course of numerous passages *in vitro* comes as unexpectedly. This suggests that CAFs could go through either genetic or epigenetic changes. Cancer-associated fibroblasts typically secrete matrix metalloproteinases (MMPs), inhibitors of matrix metalloproteinases, and extracellular matrix (ECM) components to modulate various elements within the tumor microenvironment (24).

RETRACTED

MicroRNAs, also known as miRNAs, are a type of small RNA that play a crucial role in posttranscriptional gene regulation. They are non-coding in nature and are considered to be the primary participants in this process. They play a role in both physiologically normal and pathologically induced circumstances. Numerous studies have shown that, in addition to different proteins encoded by genes, miRNAs may operate as tumor suppressors or promoters to regulate tumor behavior. MiRNAs can control various parts of cancer biology, including tumor growth and spread, resistance to immune attack, stem cell maintenance, metabolic reprogramming, and angiogenesis (25). The specialized cell types inside the tumor microenvironment should be researched separately to get a deeper understanding of cancer biology, since malignant tumors are now widely understood to be complex pathological organs. Prior research has shown that cancer cells may alter the expression patterns of miRNAs in the tumor microenvironment to influence stromal cells. Also, circulating miRNAs have been identified as biomarkers for early cancer identification and treatment outcome prediction. Evidence is mounting that tumor cells secrete micro vesicles containing miRNAs in order to connect with stromal cells in their immediate surroundings or in distant organs. Micro vesicles deliver these miRNAs to their intended stromal cells, where they act as messengers and direct them to promote tumor growth and spread (26).

## 3 Types and stages involved in prostate cancer

Prostate cancer is a deadly disease with symptoms that don’t always show up right away. It has been broken down into two different types by scientists. One is called aggressive cancer because it spreads quickly, and the other is called non-aggressive cancer because it spreads slowly.

### 3.1 Types on the basis of molecular characterization

#### 3.1.1 Primary prostate cancer

Ninety percent of prostate cancer patients had localized disease when they were diagnosed (27). The significant genomic heterogeneity of primary prostate cancer is shown by the wide variation in the clinical response to treatment in these patients (28). The ability to categorize this diverse illness into subgroups distinguished by changes in the epigenetic, transcriptomic, and complete set of human genes that make up the genome makeup of tumors has been made possible by advancements in Next-Generation Sequencing (NGS) technology. It’s crucial to note that significant additional functional genetic alterations result from structural alterations, such as gene fusions from the ETS family in the genome (29). Connected to the TMPRSS2-ERG combination status of tumors are notable differences in DNA methylation patterns, cistrome (including histone acetylation H3K27ac), and transcriptome (30). There are several other methods for categorizing prostate cancer. Instead of defining driving genetic abnormalities, they draw encouragement from tumors of the breast and additional forms of carcinoma, where distinctive transcriptional profiles continue to exist and are utilized for prognostication and therapy decision-making (31, 32). Gene expression may be classified using the well-known PAM50 marker that was recently used in the cure of prostate cancer. The classifier is often employed in the diagnosis of breast cancer’s several molecular subtypes (33).

RETRACTED

Since oncogenic pathways share so many similarities with those in breast cancer, it is not surprising that this feature can reliably categorize fatal prostate cancer (34). The PAM50 classification was used to divide prostate cancers into three groups: basal, luminal A, and luminal B. Regardless of established clinicopathological factors, they differ in clinical prognosis (35, 36). Despite using a different strategy, other transcriptomics categorization efforts reliably discriminate between luminal and basal groupings. The relationship between hormone signaling and prostate cancer categorization is particularly intriguing for predicting ADT response and/or choosing individuals for adjuvant treatment.

#### 3.1.2 Advanced prostate cancer

Modern advancements have not stopped deadly prostate cancer metastasis from occurring. Understanding the complex genetic makeup of metastatic prostate cancer has led to the development of new therapeutic approaches (28). Prostate cancer that has progressed following androgen deprivation therapy to CRPC is still reliant on androgen signaling, except in rare situations of neuroendocrine differentiation. These findings explain why AR aberrations (mutations and amplification) are so prevalent in CRPC but not in primary tumors (29). In CRPC, the expression of AR cofactors, chromatin modifiers, and transcriptional coactivators is altered, which requires RNA sequencing for precise analysis (37). The understanding and molecular study of lethal prostate cancer is being developed through genomic technologies, which also provide proper identification through the multi-modified actionable protocols of CRPC. Which directly include the pathways PI3K/AKT/mTOR and also DDR (38). And the drugs targeting the involved pathways in prostate cancer are evaluated in CRPC patients. The increase in the use of powerful anti-androgens like enzalutamide and androgen production inhibitors like abiraterone acetate while dealing with late-stage prostate cancer increases the treatment of something called double-negative CRPC. This particular group did not show characteristics of neuroendocrine as it is independent of androgen signaling (39). On the basis of limited patient numbers, genomic research shows that the development of changes in recognized prostate cancer genes is not a factor in the progression of this double-negative phenotype (40). Effectiveness of particular inhibitors *in vivo* and *in vitro* has been shown in double-negative prostate cancer models, and these tumors usually display active FGF receptor and MAPK signaling to avoid the AR pathway, resulting in delayed prostate cancer progression. Last but not least, expression profiling has also been used to identify subgroups of prostate cancer bone metastases. Here, two groups were characterized, one with the opposite characteristics (low immunological response, high metabolic activity, and high AR). All things considered, these innovative molecular stratification approaches for subgroups of patients with advanced prostate cancer have the potential to considerably benefit patients in choosing the optimum course of therapy, eventually improving quality of life and overall survival.

RETRACTED

### 3.2 Stages of prostate cancer

The staging is a way for doctors to figure out how far prostate cancer has spread in a person’s body and how it has spread to other parts of the body (41). Doctors figure out the stage of cancer based on TNM. The PSA level and Gleason score are also important (42). In TNM, T stands for “tumor,” which tells the size of the primary tumor and also its location in the prostate. N stands for “node,” which illustrates the cancer cells that have metastasized to the lymph nodes. If so, where and how exactly? M stands for “metastasis”, which tells whether and how much prostate cancer has spread. Then Gleason X says that Gleason’s score is undetermined. Gleason 6 and lower tell about the well-differentiated cells that are seen. Gleason 7 elaborates on the moderately developed cells, seeing healthy cells. And Gleason 8, 9, or 10 state that the cells have a highly distinct appearance compared to healthy cells; these cells are referred to as poorly differentiated or undifferentiated cells.

Stages are I, II, III, and IV. Which are also subdivided on the basis of their behavior and biological manner.

**Stage I**: When detected at this stage, cancer often progresses slowly. Apart from just affecting one side of the prostate, the tumor is so small that it is undetectable (or even a smaller portion than that). There hasn’t been much of a rise in PSA. Cancerous cells mimic healthy ones outside.

**Stage II:** The prostate is the only organ in which the tumor is discovered. The level of PSA is either medium or low. The prostate cancer at stage II has not yet progressed outside the prostate, but there is a rising possibility that it will. There are three distinct categories within Stage II, as follows:

**Stage IIA:** The tumor only affects a small area on one side of the prostate, making it impossible to feel. The PSA levels are around average, and the cancer cells are well differentiated. In addition, bigger tumors that are solely present in the prostate are included when the cancer cells are very different from each other.

**Stage IIB:** The tumor is contained entirely inside the prostate, making DRE detection possible if large enough. This level of PSA is intermediate. Little amounts of differentiation may be seen in the cancer cells.

**Stage IIC:** As the tumor is contained entirely inside the prostate, it may be large enough to be detected by a DRE. This level of PSA is intermediate. It is possible that the cancer cells are only partially or poorly differentiated.

**Stage III:** Higher than normal PSA values may indicate tumor progression or an advanced stage of cancer. These indicators together suggest the presence of a cancer that has advanced to the local stage and is very likely to metastasize. There are three distinct stages within III: IIIA, IIIB, and IIIC.

**Stage IIIA:** The cancer has moved from the outside of the prostate to the tissue around it. It’s possible that the seminal vesicles have been affected as well. Overall, the PSA level is rather high.

**Stage IIIB:** The cancer has probably spread beyond the prostate gland and is now invading other organs and tissues, possibly including the bladder and the rectum.

**Stage IIIC: poorly** differentiated cancer cells in the tumor seem different from healthy ones.

**Stage IV:** The prostate cancer has metastasized. The two subgroups are IVA and IVB.

**Stage IVA:** It has been determined that the cancer has progressed to the lymph nodes in the region.

RETRACTED

**Stage IVB:** It is possible that the cancer has progressed to lymph nodes farther away, as well as to other regions of the body or to the bones.

### 3.3 Prostate cancer genomics

Evolutionary processes and the underlying biology behind prostate cancer drive it towards the advanced version of the disease; this has been stated via studies that inspect the alterations to the genome involved in prostate cancer from autopsy samples (43). To analyze the metastatic site biopsies, results, and tests of the living CRPC patient’s survival, whole transcriptome sequencing (WTS) and whole-exome sequencing (WES) were performed. In contrast to localized prostate cancer, there are many mutations that may be addressed and are identified as indicating therapeutic resistance or having prognostic or diagnostic relevance (44). Seventy percent of the population has a mutation that can be targeted, and some of these mutations have been linked to ongoing clinical research (45).

## 4 Signaling pathways involved in prostate cancer

### 4.1 Pathways

Androgen deprivation therapy and therapy that targets the androgen receptor are the most promising and standard ways to treat prostate cancer (46). Both the therapies are effective in an efficient manner as they are localized to the prostate; also, the metastatic disease is castration- and androgen-sensitive in its early stages (47). To promote development and growth, the tumor seriously relies on systemic/circulating androgens to activate AR signaling. With time, the tumor itself grows to a particular stage, which is resistant, as the effect of AR and ADT antagonists is abolished (48). Tumors are more aggressive because of their adaptable nature, which allows them to use other pathways and rely less on AR signaling (48). All this aggressive behavior of tumor cells includes the overly activated PI3K-AKT-mTOR pathway (30). It is an essential signal that counteracts the inhibition of AR signaling by modulating cellular pro-survival and anti-apoptotic pathways (49). Molecular signaling pathway inhibitors and mechanism of action has been given in **Table 1**.

**Table 1:** Molecular signaling pathway inhibitors and mechanism of action.

Sr. No.	Molecular Signaling pathway inhibitors	Drugs	Brand Name	Mechanism of Action	Therapy involvement	Trial
1	Androgen Receptor signaling Inhibitor	Abiraterone	Zytiga	Reduces androgen production by blocking the enzyme, cytochrome P450 17 alpha-hydroxylase (CYP17).	Endocrine Therapy	3rd phase trial (50–52)
		Enzalutamide	Xtandi	Prevents the translocation of the AR from the cytoplasm to the nucleus. Within the nucleus, it inhibits AR binding to chromosomal DNA, which prevents further transcription of tumor genes.	Endocrine Therapy	2^nd^,3^rd^ phase trial (52–54)
		Apalutamide	Erleada	Directly inhibiting the AR at the ligand-binding domain.		2^nd^ phase trial (55, 56)
		Darolutamide	Nubeqa	Compete with androgens for binding to the androgen receptor, which reduces the ability of androgens to promote the growth of prostate cancer cells.	Endocrine Therapy	2^nd^,3^rd^ phase trial (57, 58)
2	AR inhibitors	Bicalutamide	Casodex	Binds to AR’s LBD and inhibits androgen binding. Lowers the serum level of PSA and prostate cancer symptoms.		2nd phase trial (59)
		Flutamide	Eulexin			(60)
		Nilutamide	Nilandron and Anandron			(61)
3	Poly (ADP-ribose) Polymerase Inhibitor	Olaparib	Lynparza	Inhibits poly (ADP‐ribose) polymerase, thereby blocking the repair of single‐strand DNA breaks.	Antineoplastic agents	present in 2/3 trial phase for mCRPC. (50, 62–64)
		Rucaparib	Rubraca	Inhibiting poly (ADP-ribose) polymerase, an enzyme that plays a role in DNA repair.	Antineoplastic agents	
		Talazoparib	Talzenna	Inhibition of PARP1/2 enzymes.		

RETRACTED

#### 4.1.1 Androgen receptor pathway

AR signaling is an extremely important component in both the formation and the operation of the prostate (65). Most metastatic prostate cancer and primary prostate cancer involve genetic changes in the androgen signaling system, according to the research. Castration-resistance-inducing changes include AR amplifications or mutations, an increase in NCOA1/2, and a decrease in NCOR1/2. One-third of mCRPC tumors had AR genomic structural rearrangements, which caused aberrant production of different AR variant species missing the ligand-binding domain and prolonged activation of AR signaling, such as AR variant 7 (AR-V7), which seems to promote disease development (66). In 3–4% of untreated localized prostate cancer and mCRPC cases, FOXA1 mutations inhibit androgen signaling and increase tumor development (67). Changes in the androgen receptor and related pathways are a common topic of research in metastatic CRPC. Although androgen levels are low, the AR can still be activated in CRPC through a number of different pathways (66). AR over expressed, altered androgen production, AR activating mutations, indirect AR activation, and are examples of these processes. 34% of CRPC patients had just AR mutations, which may affect their sensitivity to androgen receptor-directed treatment (67). This is because the androgen receptor mutation remains the sole clinically relevant mutation in 34% of CRPC patients. Certain androgen receptor mutations may predict responsiveness or resistance to various medicines, but their clinical importance is unknown (68). Enzalutamide and abiraterone are promising androgen receptor-targeting medicines, but most patients develop resistance to them (69). Recently, transcriptome data showed that individuals with androgen receptor V7 splice variation may react with galeterone and be resistant to enzalutamide, a new androgen receptor treatment in phase III trials, possibly proving the first treatment for CRPC based on genetic analysis. Many experimental therapies are now targeting the AR or its pathway in innovative manner, which might increase the capability to block this dominant pathway in patients with malignancies still rely only on AR signaling.

RETRACTED

#### 4.1.2 Phosphatidylinositol-3-kinase or PI3K signaling pathway

The PI3K pathway is generally activated after the stimulation of growth factor (14). Which itself triggers the signaling cascade and causes the activation of the protein kinase AKT through the phosphorylation of mTOR complex 2 (mTORC 2) and phosphoinositide-dependent kinase 1 (PDK1). The activation of AKT makes cells survive, as does the progression of the cell cycle and the proliferation via downstream effectors (70). Moreover, mTOR is a serine/threonine kinase and is a catalytic component of TORC1 and TORC2 (71). AKT-mediated suppression of TSC activates TORC1, which is a significant downstream effector. Cellular expansion and proliferation are induced when TORC is activated (71). A wide variety of human malignancies have been shown to have abnormalities in the PI3K pathway (72). In situations of advanced prostate cancer, the PI3K pathway may be dysregulated in up to 70% to 100% of cases. The PI3K pathway is negatively regulated by the protein Phosphate and Tensin Homologue (PTEN). It has been demonstrated that PTEN loss or inactivation speeds up the development of castration-resistant prostate cancer (68). Another frequent aberration found in a variety of malignancies is PI3K mutation or amplification, notably of the p110 alpha catalytic subunit (71). In regard to androgen receptor signaling, PI3K signaling interacts with it significantly (73). Pharmacologic PI3K inhibition has been linked to the activation of genes relevant to AR, according to *in vitro* research. On the other hand, AR suppression increased AKT signaling (a downstream effector of PI3K). It has been proposed that androgen suppression may favor cancers with activated PI3K pathways (71). Hence, enhanced tumor regression may result from the combination of AR deprivation and PI3K pathway suppression. In 49% of patients, the PI3K pathway was changed, following the androgen receptor, it is the most often modified pathway. Several PI3K monotherapies in the previous have been ineffective, which was assumed to be caused by coexisting changes, a lack of specificity, and signaling feedback. Clinical studies for several inhibitors of certain PI3K isoforms have been started, which may increase the specificity of these drugs (74). Recurrent PIK3CB mutations and common PTEN loss in CRPC may activate PIK3CB rather than PIK3CA, highlighting the necessity for these particular PI3K isoform inhibitors to clinically target this pathway. In addition to this, there is evidence that the PI3K pathway and the homologous recombination route interact with one another in a manner that crosses over into the other pathway. This data suggests that patients who have abnormalities in their PI3K pathway may also react to PARP inhibitors (75).

RETRACTED

#### 4.1.3 AKT pathway

AKT is the PI3K kinase’s best-known downstream effector. and is a member of the serine/threonine protein kinase family. Nevertheless, AKT may also be triggered by other kinases that are not reliant on PI3K signaling (**Figure 2**). These kinases include IKK, TANK-binding kinase 1, ACK1, SRC, ATM, and DNA-dependent protein kinase, which suggests that tumor cells have several instances of cross-talk scenarios (48). It has been shown that activation of the AKT pathway drives the establishment of PCa *in vivo* (76). In addition, phospho-proteomic analysis revealed that AKT was frequently identified as being active in samples of malignant tumors obtained through rapid autopsy. When phosphorylation occurs at both Ser473 and Thr308 sites on AKT, the protein is said to be fully activated. Nevertheless, phosphorylation at each location on its own is adequate for AKT to partly influence a fraction of subsequent cellular signaling if it is performed alone. The phosphorylation of a number of different targets by active AKT controls a number of different cellular activities. The activity of AKT is linked to transcription, regulation of protein synthesis, apoptosis, cell survival, autophagy, proliferation, and metabolism via these downstream effectors.

**Figure 2:** Illustration of signaling pathways involved in prostate cancer where PI3K and AKT pathways are shown.

#### 4.1.4 mTOR pathway

mTOR, also known as the mammalian target of rapamycin, is a serine/threonine protein kinase that is one of the most important downstream effectors of the AKT signaling pathway (77). It is interesting to note that samples of prostate cancer had greater levels of mTOR expression compared to those of benign tissue (78). mTOR is involved in interactions with a variety of proteins, which leads to the formation of two separate complexes. mTORC1 is responsive to the inhibition caused by Rapamycin, but mTORC2 is not sensitive to this kind of inhibition. Activation of mTORC1 signaling begins with AKT-mediated phosphorylation of TSC2, which suppresses the TSC1/2 complex and ultimately activates the GTP-bound RHEB, a mTORC1 activator (48). In addition, AKT-mediated phosphorylation suppresses the mTORC1 repressor PRAS40 (also present in the complex) (79). In addition to mTORC1, the AMP-activated protein kinase (AMPK), glycogen synthase kinase 3 (GSK3), and Wnt (growth factor) signaling pathways may also control TSC2. Phosphorylation and activation of p70S6 kinase (p70S6K) and inhibition of 4EBP1 both have a role in the primary biological activity that is regulated by an active mTORC1 signal. PI3K, RAS, AMPK, WNT, TSC1/2, and p70S6K are some of the proteins that have the ability to control how active mTORC2 is. Importantly, the reduction of mTORC2 activity by p70S6K results in negative feedback control of the PI3K-AKT pathway (48). This is because mTORC2 enhances AKT activation by phosphorylating Ser473, and p70S6K is responsible for this regulation. In contrast to the biological processes that are regulated by mTORC1, active mTORC2 has the ability to phosphorylate a number of downstream effectors, which in turn leads to cell survival, advancement through the cell cycle, and actin remodeling. In addition to this, it has been hypothesized that mTORC2 is essential for the formation of PCa in the absence of PTEN (80). In accordance with this, the suppression of PDK1 did not reverse greater PCa development in PTEN-deficient transgenic mice, which may indicate the likelihood of mTORC2-mediated AKT activation and/or the activation of compensatory cascades.

RETRACTED

#### 4.1.5 Role of NGF/TrkA or neurotrophins

Prostate transformation and PC development are driven by receptor tyrosine kinases (RTKs). The tropomyosin receptor kinase A (TrkA) is known to interact with nerve growth factor (NGF), leading to the activation of various signaling pathways such as Ras/mitogen-activated protein kinase (MAPK), phosphoinositide 3-kinases (PI3-K), and phospholipase C gamma (PLCγ). These pathways are responsible for promoting cell survival, proliferation, and invasiveness (81). NGF is abundantly released by the human prostate and plays a crucial role in regulating the normal development of prostate tissue. Stromal cells are known to secrete nerve growth factor (NGF), which subsequently binds to TrkA and p75NTR receptors expressed in the epithelial counterpart, thereby promoting its growth. Additionally, preliminary investigations conducted on animal models have underscored the significance of NGF/TrkA signaling in the proliferation and metastasis of prostate cancer. The production of NGF through paracrine and/or autocrine mechanisms is stimulated by molecular alterations in epithelial or stromal cells, thereby facilitating the development of prostate cancer. In addition, a frequent observation in patients with prostate cancer is the enduring manifestation of TrkA, coupled with the absence of p75NTR receptor expression. Therefore, it is possible that PC cells rely solely on the signaling pathway of nerve growth factor for their survival. It has been demonstrated in recent studies that the interaction between TrkA and AR has a significant impact on the effects of NGF in various cell types. The present study reveals that the interaction under investigation exerts regulatory control over the process of androgen-induced differentiation in neuronal-derived cells (82). Additionally, it exerts regulatory control over the processes of NGF-induced proliferation and migration in androgen-sensitive LNCaP cells. Thus, TrkA emerges as a potentially viable biomarker for drug targeting in prostate proliferative disorders. In spite of the growing body of evidence, the precise mechanism(s) responsible for the disruption of TrkA signaling in CRPC is still inadequately accepted. Furthermore, genetic screening failed to detect TrkA mutations or Trk-fusion onco-proteins in patients with prostate cancer. The results mentioned previously provide additional support to the notion that disruption of a functional NGF/TrkA signaling pathway could potentially play a role in the advancement of prostate cancer.

RETRACTED

#### 4.1.6 DNA damage repair pathway

Alterations in the mechanisms responsible for DNA mismatch repair and homologous recombination are the most common types of DNA damage response abnormalities, and advanced prostate cancer patients have a relatively high prevalence of both types of mutations. Early clinical efforts to treat this vulnerability centered on blocking the poly ADP ribose polymerase family, which detects and repairs damaged DNA (83). These efforts were focused on limiting PARP since it plays a key role in these processes. Olaparib is an oral PARP inhibitor that was studied in men with metastatic prostate cancer that was resistant to castration (84). Positive results from phase 2 were published, and the most common side effects were anemia and being tired. People with breast cancer susceptibility, BRCA 1 or 2 mutations or ataxia telangiectasia serine/threonine kinase (ATM) mutations, which are all important parts of DNA repair pathways, often respond better to treatment than those without these mutations. According to other results that were published not too long ago, the loss of the chromatin remodeler chromodomain-helicase-DNA-binding protein 1 (CHD1), which is often seen in advanced prostate cancer, is associated with an increase in the responsiveness to PARP inhibitors. The positive clinical phase 2 findings that were achieved with olaparib led to a breakthrough designation being granted by the FDA, and a phase 3 pivotal trial is presently being conducted. In contrast, the clinical data obtained for the PARP inhibitor veliparib administered to patients with metastatic castration-resistant prostate cancer in conjunction with abiraterone acetate did not demonstrate a statistically meaningful improvement (85). Inhibition of the enzyme known as ataxia telangiectasia and Rad3-related kinase, which detects breaks in single-stranded DNA, is still another strategy. In a bone metastasis xenograft model of CRPC, it was shown that the ATR inhibitor BAY 1895344, when used in conjunction with radium-223 dichloride, had significant anti-tumor activity. Chk1 is a cell-cycle regulator that is downstream of ATR in the DNA damage response, and new results reveal that its inhibitor, AZD7762, is additive or synergistic with enzalutamide in prostate cancer xenografts (86). Despite this, clinical investigations with this molecule have been halted.

RETRACTED

### 4.2 Inhibitors of signaling pathways

Numerous studies have demonstrated the progression of prostate cancer pathways wherein PI3K/mTOR/AKT signaling pathways have proved to play a crucial role. PTEN (the phosphatase that directly opposes the oncogenic signaling pathways) loss is the major or crucial step due to which the event of PI3K signaling gets hyperactive, and it’s connected with the negative result in the patient with prostate cancer. The stages observed in humans can be easily observed in the transgenic mouse model with the specific prostate gene deletion of the PTEN gene (87). The mechanism of reciprocal feedback between AR signaling and the PI3K/AKT/mTOR pathway has been noticed (**Figure 2**). PI3K pathway inhibition is one reason an increment in the level of AR protein occurred, which also restores AR signaling (87). The PI3K/mTOR/AKT pathway inhibitors exhibit anti-tumor activity in *in-vivo* experiments in several preclinical studies, and the AR antagonist has a comparable anti-tumor effect. Clinical research on the PI3K/mTOR/AKT pathway has produced positive outcomes in some patterns of activity. Ipatasertib is an AKT inhibitor recently in phase 3 clinical trials for patients with mCRPC (88). The different combinations are being implicated with enzalutamide or abiraterone acetate in some trials, but the results of the first phase 2 were not promising. Better outcomes were expected based on the mutations in the patient hierarchy in the pathways PI3K/mTOR/AKT and PTEN loss. Variations have been reported in almost every subgroup pertinent to a substantial percentage of patients, in early-stage tumors, and consequently, in metastases. Pathways such as the PI3K/AKT/mTOR pathway’s inhibitor with limited response may be further linked to the activation of the compensatory cascade of mitogen-activated protein kinase (MAPK), and the relevant research using preclinical models of prostate cancer demonstrates that the cancer is increasing enormously after blocking both channels together (89). Trametinib, a MEK (MAPK kinase) inhibitor and a component of the MAPK pathway upstream, is now being tested in late-stage prostate cancer clinical trials. Prostate cancer, particularly late-stage disease, has been reported with the vital role of fibroblast growth factor signaling (90). Different clinical trials are running in an alternative manner with different therapeutics and combinations of drugs, whereas no dedicated trial has been addressed yet, especially for prostate cancer.

RETRACTED

## 5 Diagnostics for prostate cancer

Diagnostics for prostate cancer are themselves a constantly changing specific area that performs a crucial and essential role as it ensures a suitable and appropriate therapeutic course for the patient, which also prevents them from overdiagnosis and overtreatment (91). Digital rectal examination and detection of serum prostate specific antigen continue to raise suspicion of prostate cancer despite the many advancements in the area (92). Then, in order to properly educate patients on the dangers and advantages of a prostate biopsy, urine biomarkers, additional derivatives of blood PSA, and multiparametric magnetic resonance imaging can assist in risk stratifying individuals (93). A range of imaging modalities, including bone scintigraphy, CT scan, can be used to further stage prostate cancer after a diagnosis is made (**Figure 3**).

**Figure 3:** Illustrates a variety of diagnostic procedures, including both primary and more sophisticated forms of diagnostics.

### 5.1 Imaging

Imaging is rapidly evolving as a diagnostic for prostate cancer, as it can provide images of a particular area of the prostate, which can also help to identify the type and stage of cancer. This will also help to avoid unnecessary biopsies.

### 5.2 Digital rectal examination

A digital rectal examination is a diagnostic tool that is specifically used to check the prostate for the disease called cancer and also gives the measurements of the prostate by >0.2 mL. It can also test for prostate specific antigen. DRE can also go for a high degree of interobserver variability (94). The chance of severe prostate cancer is still present despite DRE. According to a historical prospective multicenter investigation, DRE detected 18% of prostate cancers. Regardless of the PSA, a prostate biopsy is still recommended if the DRE is abnormal (95).

RETRACTED

### 5.3 Transrectal ultrasound

A hypoechoic lesion on a standard B-mode transrectal ultrasound may represent prostate cancer, which is non-specific conclusion (96). A significant difference was not identified in the prostate cancer detection rate from biopsies of individuals with or without hypoechoic lesions (25.5% versus 25.4%), according to large prospective research (97). This demonstrates that a hypoechoic lesion alone does not correlate with a rise in the incidence of cancer and B-mode transrectal ultrasound by alone cannot diagnose prostate cancer (98). Even though, it is essential for locating the prostate in order to take biopsies (99). The analytical rate of additional ultrasound imaging alterations for the recognition of prostate cancer has also been examined (100). Due to the increased tumor vasculature, color doppler ultrasound (CDUS), which monitors blood flow, may be able to identify prostate cancer (101). When used with the standard B-mode transrectal ultrasonography, color doppler ultrasound worked best in high-grade illness and early evaluations of the technology revealed it could detect up to 70% of prostate malignancies. However, second research found that when compared to normal transrectal ultrasonography, the use of color doppler ultrasound in targeted prostate biopsies did not increase prostate cancer detection rates (102). To identify enlarged microvasculature in the prostate, contrast-enhanced ultrasonography (CEUS) involves microbubble contrast agents. When compared to unenhanced color doppler ultrasound, it has been found to increase sensitivity in the detection of prostate cancer (97). The foundation of sono-elastography is basically the idea of elastic characteristics of normal and cancerous prostate tissue that differ significantly. Doppler ultrasonography is used in the method to find regions of aberrant stiffness by estimating the response of tissues to harmonic mechanical stimulation (103). Sono-elastography was reported to be capable of detecting 84.1% of prostate tumors in the initial research looking at its application. While each of these three methods has showed potential in preliminary research to increase prostate cancer diagnosis, combination imaging is reportedly the most advantageous (104). B-mode, sonoelastography, and contrast-enhanced ultrasonography (CEUS) together make up Multiparametric ultrasonography (mpUS), which increased the sensitivity for clinically relevant prostate cancer to 74% from 55%, 55%, and 59%, respectively. However, there is uncertainty about the use of ultrasonography in the diagnosis of prostate cancer, particularly with the new development of multiparametric-MRI (mp-MRI), which is further precise than Multiparametric ultrasound (mp-US). The unique ultrasound method that has potential to challenge mp-MRI is micro-ultrasound. In contrast to the newer modality of micro ultrasound, which works at a frequency of 29 MHz, traditional TRUS uses frequencies of 6–9 MHz (98). This provides a 300% increase in picture resolution, enabling the identification of minute alterations in ductal structure. Early results have shown that this method is more effective at detecting clinically relevant prostate cancer and might be find lesions that multiparametric-MRI was unable to find. But further study is needed to determine the precise function that micro-ultrasound will play for the result of prostate cancer.

RETRACTED

### 5.4 Multiparametric magnetic resonance imaging

The European Association of Radiology of the Urinary Tract advises using high-resolution T2 weighted images in conjunction with multiparametric MRI to identify prostate cancer, Dynamic contrast enhanced (DCE) imaging and diffusion weighted imaging (DWI) are at least two functional MRI approaches. T2-weighted MRI typically shows a round low signal intensity focus, high signal intensity on DWI at high b-values, and traditionally shows premature improvement on DCE-MRI as the typical signs of prostate cancer (105). Each lesion is given a score between 1 and 5 that forecasts its likelihood of existence a clinically significant prostate cancer, with 5 indicating a very high likelihood (106). This system, called the Prostate Imaging-Reporting and Data System (PI-RADS), offers a structured way to report each lesion. According to a meta-analysis evaluating the mp-diagnostic MRI’s efficacy for prostate cancer, it has high specificity and sensitivity, 88% and 74%, respectively, and a varied but high negative predictive value, 65-94%. Additionally, a comparison between radical prostatectomy histology and pre-operative MRI revealed that the likelihood of detecting prostate cancer grew with both tumor volume and rising Gleason score (107). Finding a target for a biopsy to increase the identification of clinically relevant prostate tumors is one of the primary uses of mp-MRI. Moreover, a prebiopsy mp-MRI can be utilized to prevent performing biopsies on individuals who have no apparent lesions. According to the PROMIS experiment, 27% of patients might have avoided a biopsy by utilizing an mp-MRI and only conducting a prostate biopsy on patients with PI-RADS lesions of less than three (108).

### 5.5 Computed tomography

Computed tomography has been demonstrated to be an unreliable technique for the detection of lymph node metastases (109). A meta-analysis discovered an excellent specificity of 82% but a low sensitivity of 42% for mp-MRI (57). Due to their dependence on nodal enlargement, which is not always present, CT and mp-MRI have significant limitations in their ability to identify lymph node metastases. The data from CTs can be used to categorize prostate cancer.

RETRACTED

### 5.6 Advancements techniques

#### 5.6.1 Choline positron emission tomography CT

Choline Positron Emission Tomography (PET) CT rely on the increased radiotracer uptake that is considered to be caused by an rise in membrane phosphatidylcholine in cancer cells (110). Its utility in diagnosing prostate cancer has mostly been examined for its capacity to identify lymph node metastases, with mixed findings. Nevertheless, its application in high-risk prostate cancer has shown a noticeably enhanced specificity and sensitivity, indicating that it may be helpful in these circumstances for the identification of nodal metastases (111). It is uncertain, that whether choline PET-CT will play a part in the future of prostate cancer diagnostics given the advancements in 68Gallium (68Ga) labelled prostate specific membrane antigen PET-CT.

#### 5.6.2 Bone scan

CRPC patients concern about bone metastases. Radium 223, bisphosphonates, and the RANKL inhibitor denosumab treat bone metastases (112). The most common method of detecting bone metastases is a technetium Tc 99m methylene disphophonate (Tc 99m MDP) bone scan (113). Clinical stage, Gleason score, and PSA are all highly reliable indicators of bone metastases. Patients with intermediate-risk (PSA 10–20 ng/ml or Gleason score 7 or cT2b) or high-risk (PSA >20 ng/ml or Gleason score 8–10 or cT2c/3/4) prostate cancer are advised to have a staging baseline bone scan. These criteria were shown to have a negative predictive value of 99.6%, meaning that roughly 81% of patients wouldn’t need to undergo staging with a baseline bone scan (114). Clinical trials are validating genetic changes in DNA repair mechanisms. Olaparib, rucaparib, and talazoparib are being tested in phase 2/3 studies for metastatic castration-resistant prostate cancer (115). Early clinical trials on immune checkpoint inhibitors including CTLA4, PD1, and PD-L1 have also been conducted. The expression of prostate-specific membrane antigen (PSMA) is notably elevated in the cell membranes of prostate cancer. Several clinical studies have assessed the efficacy of small molecules or antibodies targeting PSMA and labelled with radionuclides or cytostatic agents. In addition, a wide range of pathways related to cell growth and survival, such as the PI3K/AKT/mTOR pathway, exhibit interaction with androgen receptor signaling, and contribute to the advancement of prostate cancer. Clinical studies have explored the efficacy of PI3K/AKT/mTOR specific inhibitors as a monotherapy, as well as combination therapies with AR signaling inhibitors (116). Epigenetic modifications, including but not limited to histone methylation and acetylation, as well as DNA methylation, are widely observed in cases of prostate cancer.

RETRACTED

#### 5.6.3 Prostate specific membrane antigen-based (PET/CT)

It’s very promising that 68Ga PSMA PET-CT will enhance the detection of prostate cancer (117). Nearly all prostate cancer cells have excessive PSMA expression on their cell membranes (118), and the expression levels change depending on the tumor’s stage and grade. In a meta-analysis, 68Ga PSMA PET CT was reported to have a better sensitivity (65% versus 41%) than MRI for the detection of lymph node metastases in individuals with intermediate or high-risk prostate cancer. In comparison to choline PET-CT, MRI, and bone scintigraphy, a subsequent meta-analysis has shown that 68Ga PSMA PET-CT had the greatest sensitivity and specificity for the diagnosis of bone metastases (119). Another recent multicenter randomized trial discovered that 68Ga PSMA PET-CT had a 92% accuracy rate and was superior to bone scan and CT in males with high-risk prostate cancer (Gleason grading group 3-5, PSA 20, or clinical stage T3). The patient’s care plan had to be altered more frequently as a result of the enhanced staging strategy, which is significant since it might potentially provide the best first-line therapy while also preventing unneeded treatment.

## 6 Therapeutics

### 6.1 Current therapeutic approaches

The primary and successful therapeutic target continue to exist is the androgen receptor (120). AR finding, including the mechanism of AR resistance has qualifies several productive treatments in the patient of CRPC. In this space, we have approved therapies includes new agents of a pathway of androgen synthesis, such as abiraterone (121). Enzalutamide as androgen receptor’s direct inhibitor (122). In spite of that, the major patients of CRPC develops the resistance towards the focused therapies of androgen receptor. Also, many more patients had never respond to the therapies. Generally, the major ratio of patients of CRPC, eventually succumb to the disease.

### 6.2 Science-driven development of therapeutics

For new genes in prostate cancer, the novelty of quick and sophisticated computational techniques to applications has been investigated and will continue to be investigated. Through gene expression analysis, the translocation of the TMPRSS2-ERG gene was identified. The Genome is itself a complete regulatory network (interactome) through which human and mouse gene is easily access-able to search for a particular gene. For prostate cancer malignancy, FOXM1 and CENPF are synergistic master of regulators. Whereas, the drug designed as singular and in combinations will ensure to inhibit the carcinogenic activity or the malignancy of FOXM1 and CENPF (123). In the treatment of other cancer types, monotherapy and combination therapy are successfully used (124). Likewise, effective therapies are yet to emerge out for prostate cancer. Novel combination techniques have been developed as a result of mechanistic preclinical investigations, and they have sparked a number of clinical studies aimed at the treatment of prostate cancer (125). Status of Ongoing clinical trials of potential medications in CRPC advanced stage patients. has been given in **Table 2**.

RETRACTED

**Table 2:** Status of Ongoing clinical trials of potential medications in CRPC advanced stage patients.

SR.NO.	TARGETS	CUURRENT CLINICAL TRIALS/THERAPIES	POTENTIAL THERAPEUTIC	PHASES
1.	Androgen Receptor	NCT01162395	AZD3514	Primary
		NCT00186108	Triamcinalone	Primary
		NCT00140478	Mifepristone (RU-486)	Secondary
		NCT01615120	GTx-758	Secondary
		NCT02445976	VT-464	Secondary
		NCT00181597	Trilostane	Secondary
		NCT02012296	Mifepristone/enzalutamide	Primary and Secondary
		NCT00569153 NCT01809691 NCT01809691	Orteronel (TAK-700)	Primary, Secondary, and Tertiary.
		NCT02438007	Galeterone	Tertiary
2	Immunotherapy	NCT02411786	AR DNA Vaccine	Primary
			BNIT-PR-001	Primary
		NCT00170157	Ipilimimab	Secondary
		NCT01377389	pilimimab þ ADT	Secondary
3	PIK3CA	NCT02487823	Buparlisib (BKM120)	Primary
	PIK3CB	NCT01884285	AZD8186	Primary
	PIK3CB	NCT02215096	GSK2636771/enzalutamide	Primary
	PIK3CB	NCT01485861	GDC-0068/abiraterone	Secondary
4	Cell Cycle, CDK4/6	NCT02555189	Ribociclib	Primary and Secondary
	CDK4/6	NCT02059213	PD 0332991	Secondary
	BCL-2	NCT01828476	Navitoclax/abiraterone	Secondary
5	DNA damage, PARP	NCT02500901, NCT00749502	Niraparib/enzalutamide	Primary
		NCT01286987	BMN 673	Primary
		NCT00892736	Veliparib	Primary
		NCT01972217	Olaparib/enzalutamide	Secondary
6	WNT	NCT02020291	Foxy-5	Primary
		NCT01608867	OMP-54F28	Primary

Firstly, In androgen responsive tumors, the novel targeted therapies in combination with androgen signaling were explored (126). Enzalutamide may have induced a response in preclinical models when the PARP inhibitor Olaparib reduced the expression of BRCA1 in prostate cancer cells carrying wild-type BRCA1 (127). In the mCRPC patient’s clinical efficacy benefits were provided through, a randomized trial of a phase 2 olaparib in combination with abiraterone (NCT01972217) (128). PI3K inhibitors were coupled with AR inhibitors to target the mutually detrimental regulation of AKT and AR signaling in preclinical models. In human prostate cancer patients, to evaluate the efficacy of these treatments, further clinical trials are required. Protein inhibitors (GS-5829 and ZEN003694) are BET domains, which in combination with primary and secondary phase trials of enzalutamide, are currently used to target the AR cross-talk and BRD4 in mCRPC (NCT02711956 and NCT0 2607228).

RETRACTED

Secondly, in an ADT clinical trial, enzalutamide (NCT02861573) in combination with anti-PD-1 (pembrolizumab) and enzalutamide (NCT03016312) in combination with anti-PD-L1 (atezolizumab) were potentially tested to modulate the priming of tumor-specific adaptive immune responses (129).

Third, AR+ adenocarcinoma converts into small cell carcinoma or AR-independent NEPC, demonstrated via preclinical models (130). In androgen-insensitive tumors, some genes show a vital and a crucial role like as EZH2, AURKA, BRN2 (also called POU3F2), MYCN, and SOX2, monotherapy targets the gene or combination therapy with inhibitor of EZH2 (EPZ-6438 or GSK126) and in preclinical studies the therapeutic benefits were shown via enzalutamide. Targeting repair pathways of DNA damage offers the best chance for a novel prostate cancer treatment (131).

### 6.3 Chemotherapy

The advancement of therapeutic drugs, whether singular or in combination, gives promising results, whereas for the treatment of prostate cancer, certain chemotherapy medicines have received the approval of the FDA (132). To stop tubulin depolymerization, drugs called capaztaxel and docetaxel are injected intravenously every three weeks. These drugs ultimately result in cell death by preventing mitotic cell division (133). AR inhibitory characteristics have been associated with the inhibition of microtubule-dependent nuclear transport. The FDA authorized the drugs docetaxel and cabazitaxel in 2004 and 2010, respectively, for the treatment of mCRPC (134). In clinical trials for two different times, positive results were recorded for metastatic hormone sensitive prostate cancer, evaluated with docetaxel in common with ADT (135). The observed adverse effect on the frequent basis is hetpatological toxicity such as neutropenia. As compared to docetaxel, the topoisomerase inhibitor mitoxantrone, which alleviates certain symptoms, has a minor survival advantage in prostate cancer (136). Together with cabazitaxel, it produces long-lasting effects in mCRPC patients who have never had chemotherapy. The use of mitoxantrone is controlled in the presence of serious side effects (137).

### 6.4 Immunotherapy

Sipuleucel-T received clearance for mCRPC in 2010 (138). Leukapheresis has been used in immunotherapy of autologous cellular origin to make the cells, which are peripheral and mononuclear blood cells, via the patient’s body. The cells were then grown for antigen-presenting cell maturation (139). In order to convert cancerous prostate cells back into normal ones, the patients are then given the activated product, which expresses PAP at a high level, over the course of three intravenous infusion sessions. The reported side effects are for a long time as in clinical benefits were only mild and manageable. Hence, the high price and complicated technique have prevented sipuleucel-T from being used widely up to this point (140). As prostate cancer has a relatively little percentage of neoantigens particular to tumors, it has a certainty to react to a pair of immunological checkpoints inhibitor-focused therapies. The Neoantigen burden may get increased as the defects were reported in DNA repair pathways in both late and early phase (141). The microenvironment of prostate tumors is a current issue of interest because it suppresses the immune system and interferes with natural killer cell activity (141). Conducted research mostly using the models are non-tumor which suggests that the prostate microenvironment’s immune cells get influence by local sex steroids (142). The use of checkpoint inhibitors in several cancer types offers a significant survival benefit (129). In prostate cancer, evaluation of the potential benefits of immunotherapy is done (143) Ipilimumab, an antibody which is anti-CTLA4, gives beneficial results in the clinical studies with patients having prostate cancer, no enhanced overall survival could be confirmed in subsequent bigger investigations, despite the fact that full remission was achieved in a few cases. Durable responses in people with metastatic prostate cancer have previously been seen in two clinical trials looking at the anti-PD-1 antibody which is pembrolizumab (144). Most importantly, the medication pembrolizumab has achieved tissue clearance agnostic for solid tumors with a deficiency of mismatch repair, allowing this therapy to be used for patients with advanced prostate cancer (145). Metastatic prostate cancer therapy Using atezolizumab, durvalumab, and avelumab, anti-PD-L1 antibodies are being investigated in preliminary clinical studies (146). In the most recent randomized phase 3 study, atezolizumab as a single medication is compared to an amalgamation with enzalutamide (145). PD-L1 expression in tumors, anomalies in DNA repair pathways, and the use of medicines that cause genomic instability can all be used to select individuals for trials that evaluate checkpoint inhibitors. Recently, a thorough analysis of clinical trials for prostate cancer, including this class of biological chemicals, was published (147).

RETRACTED

### 6.5 Radiation therapy

In order to eradicate cancer cells or stop them from proliferating, radiation therapy employs high-energy x-rays or other forms of radiation (6). Radiation treatment comes in a variety of forms:

#### 6.5.1 External radiation therapy

External beam radiation therapy involves the utilization of an external device to deliver targeted radiation to the specific region of the body afflicted with cancer and cover the large area whereas Conformal radiation therapy is an external radiation modality that employs computerized technology to generate a three-dimensional (3D) representation of the malignant growth and also specifically customizes the radiation beams to conform to the tumor’s shape. This approach enables the delivery of a substantial radiation dose to the tumour while minimizing the impact on adjacent healthy tissue (148).

#### 6.5.2 Hypo-fractionated radiation therapy

It could be prescribed due to its more convenient treatment regimen. Hypo-fractionated radiation therapy is a modality of radiation treatment that involves the administration of a higher cumulative radiation dose over a reduced number of days, as compared to the conventional radiation therapy. The potential for increased adverse effects of hypo-fractionated radiation therapy in comparison to standard radiation therapy is based upon the specific schedules applied (149).

#### 6.5.3 Internal radiation therapy

The administration of a radioactive substance enclosed within needles, seeds, wires, or catheters that are inserted in close proximity to or directly into the cancerous area is a common practice. Radioactive seeds are typically implanted in the prostate gland during the initial stages of prostate cancer via percutaneous needle insertion through the cutaneous tissue located between the rectum and scrotum. The localization of radioactive seeds within the prostate gland is facilitated by utilizing imaging modalities such as transrectal ultrasound or computed tomography. The extraction of needles follows the insertion of radioactive seeds into the prostate.

#### 6.5.4 Radiopharmaceutical therapy

Radioactive material is utilized for the purpose of cancer treatment. The administration of therapeutic agents that emit radiation, also known as radiopharmaceutical therapy, encompasses the following:

The therapeutic approach of alpha emitter radiation involves the utilization of a radioactive material for the treatment of bone metastases in patients with prostate cancer. Radium-223, a radioactive element, is administered intravenously and subsequently circulates through the vascular system. Radium-223 exhibits the tendency to accumulate in osseous regions afflicted with neoplastic growths, thereby inducing apoptosis in the malignant cells.

RETRACTED

The modality and administration of radiation therapy are contingent upon the specific classification and progression of the neoplastic condition under consideration. The administration of radiation therapy to male patients with prostate cancer has been associated with an elevated likelihood of developing cancer in the bladder and/or gastrointestinal tract. The administration of radiation therapy has been found to be associated with the development of impotence and urinary complications, which may exhibit worsening in the extent over time.

### 6.6 Hormone therapy

Hormone therapy is a therapeutic intervention for cancer that involves the removal or inhibition of hormones, thereby hindering the proliferation of cancerous cells. Hormones are endogenous chemical messengers synthesized by specialized glands within the human body and subsequently transported throughout the circulatory system. Prostate cancer growth can be stimulated by male sex hormones. Pharmaceutical interventions such as drug therapy, surgical procedures, or hormonal treatments are employed to mitigate the effects of male hormones by either reducing their quantity or impeding their functionality. The medical intervention commonly referred to as ADT is formally known as androgen deprivation therapy (150).

Pharmacological intervention for prostate cancer may encompass the subsequent measures involving hormone therapy:

1. Antiandrogens have the ability to impede the activity of androgens, which are hormones that stimulate the development of male sexual characteristics, including testosterone. Like:- enzalutamide, darolutamide, and apalutamide.
2. Abiraterone acetate has the ability to inhibit the androgen biosynthesis pathway in prostate cancer cells. This treatment modality is indicated for males who present with progressive prostate cancer that has not responded to prior hormonal interventions.

Additionally, it is employed in males diagnosed with high-risk prostate cancer who have exhibited improvement subsequent to undergoing hormone level reduction therapies.

3. The administration of estrogens, which are known to facilitate the development of female sexual characteristics, has the potential to inhibit the production of testosterone by the testes. The use of estrogens in the management of prostate cancer is infrequent in contemporary medical practice due to the risk of crucial adverse reactions.
4. Releasing hormone agonists as Luteinizing hormone have the potential to inhibit the biosynthesis of testosterone in the testes.
5. The orchiectomy is a surgical intervention aimed at the removal of one or both testicles, which constitute the primary endocrine glands responsible for the production of male hormones, including testosterone, with the purpose of reducing the overall hormone output.
6. Pharmaceutical substances that are capable of inhibiting the synthesis of androgens by the adrenal glands are progesterone, aminoglutethimide, and ketoconazole.

RETRACTED

Men undergoing hormone therapy may experience a range of adverse effects, such as hot flashes, sexual dysfunction, reduced sexual urges, and decreased bone density. Additional adverse reactions comprise of diarrhea, nausea, and allergic reactions.

### 6.7 Targeted therapy

Targeted therapy is a therapeutic modality that employs pharmacological agents or other substances to selectively recognize and combat particular malignant cells. Compared to chemotherapy or radiation therapy, targeted therapies are known to induce comparatively lesser damage to normal cells. enzyme that participates in various cellular processes are being blocked via PARP inhibitors also the enzymes involve in DNA damage repair. Inhibiting this enzyme may aid in preventing cancer cells from repairing their damaged DNA, ultimately leading to their demise (151).

### 6.8 Bisphosphonate therapy

When cancer has spread to the bones, bisphosphonate medications like clodronate and zoledronate diminish bone disease. Men who undergo orchiectomy or antiandrogen treatment are more likely to have bone loss. Drugs called bisphosphonates lower the risk of bone fractures in these patients. Clinical trials are currently investigating the efficacy of bisphosphonate drugs in the prevention or deceleration of bone metastasis growth (152).

## 7 Future perspectives

Metastatic castration-resistant prostate cancer has been treated with several therapies. But many chemotherapies have been proven ineffective in the treatment of metastatic castration-resistant prostate cancer (153). However, docetaxel versus mitoxantrone treatment led to an improvement in the survival rate of patients, but it had the limitation of improving the survival rate only for a shorter duration of time (154). Metastatic CRPC patients have several new therapy choices because of the record number of medication approvals in the previous year. Sipuleucel-T, abiraterone acetate, cabazitaxel, and denosumab are FDA-approved drugs for the treatment of metastatic CRPC (155). Experts should highlight the challenges of using these new medicines in metastatic CRPC patients. The therapeutic and diagnostic treatments conducted in response to prostate cancer and castration-resistant prostate cancer have a large number of published reports highlighting the adverse effects on the patient’s physiology and mental state, and furthermore, they stimulate various psychological disorders.

RETRACTED

The primary therapy is chemotherapy, which uses powerful drugs to kill cancer cells or stop their growth. It can be highly effective in treating cancer, but it often comes with side effects. These side effects can vary depending on the specific drugs used, the dosage, the duration of treatment, and the individual’s overall health. Some common side effects of chemotherapy are fatigue, nausea, vomiting, hair loss, loss of appetite, weakened immune system, increased risk of bleeding and bruising, peripheral neuropathy, constipation or diarrhea, cognitive changes, etc. (156). Immunotherapy has shown promising results in treating various types of cancer, including prostate cancer, but it has also got many adverse effects. The specific adverse effects of immunotherapy for prostate cancer can vary depending on the type of immunotherapy used. Some potential adverse effects include immune-related side effects, allergic reactions, endocrine-related side effects, changes in blood cell counts, etc. (157). Afterwards, another type of therapy used is radiation therapy, which uses high-energy beams to target and kill cancer cells. Drawback of radiotherapy is that apart from targeting prostate cells, it can also affect nearby healthy tissues and organs, leading to both short-term and long-term effects. Some of the adverse effects of radiation therapy seen in case of prostate cancer patients includes skin changes, urinary problems, bowel problems, sexual dysfunction, infertility, secondary cancers, etc. (158). Likewise, another therapy is hormone therapy, also known as androgen deprivation therapy. It aims to lower the levels of male hormones, particularly testosterone, in the body or block their effects on cancer cells. Prostate cancer cells typically rely on testosterone to grow and survive, so reducing hormone levels can help slow down the progression of the disease. Some limitations of hormone therapy are that it’s not a curative treatment and typically does not eliminate cancer cells completely. Over the time, prostate cancer cells may become resistant to hormone therapy, leading to disease progression. This is known as castration-resistant prostate cancer, and additional treatment options are available for managing this stage of the disease (157). Then comes targeted therapy, which aims to selectively inhibit the growth and spread of cancer cells while minimizing damage to healthy tissues. They are generally well tolerated, but they still have side effects. Some common side effects associated with targeted therapy are skin reactions, gastrointestinal issues, increased risk of infection, changes in blood cell counts, cardiovascular effects, liver toxicity, risk of blood clots, etc. (159). Further, we have covered applications of Bisphosphonates in the treatment of prostate cancer. While bisphosphonate therapy is generally safe and well tolerated, it can have potential side effects. Some common side effects associated with bisphosphonate therapy are gastrointestinal upset, oesophageal irritation, musculoskeletal pain, and osteonecrosis of the jaw (160).

RETRACTED

The review focus on the analysis of the proteome, genome, and epigenome of prostate cancer. Furthermore, the integration of conventional chemotherapeutic medicines in conjunction with natural chemicals may potentially be a viable approach to the problem of finding a cure. Understanding the drug’s pharmacogenomics mechanisms prior to its administration to the patient may induce fewer modifications in the patient’s genome profile, thereby reducing the mentioned side effects. In addition, pharmacogenetics investigates the inherited drug metabolism and effects to find the most effective therapeutic therapy and dosage for each individual patient. This helps to minimize the adverse effects of the medical condition. Cancer therapy with chronic cytotoxicity and a component of the unpredictable are both necessary components of cancer treatment. Although genetic polymorphisms code for the metabolic enzymes and cellular targets of the majority of chemotherapy medications, after following all the protocols, it is still not possible to predict the consequences for individual patients. Understanding drug-response genetics can revolutionize several treatments. For many classes of chemotherapy agents, gene polymorphisms can predict cancer treatment outcome, but more studies in well-characterized and larger cancer populations are needed to validate pharmacogenetic markers in experimental settings before routine clinical diagnostics. However, a 100 percent effective treatment strategy has yet to be established. As for the treatment of prostate cancer in humans, large-scale clinical studies are required to assess potentially useful chemicals and determine non-toxic dosages to provide a specific treatment.

## Author contributions

Authors have contributed equally in their own right. The review was conceptualized and outlined by SQ and PS. NT worked on the idea and prepared the initial draft. SJ and BN built on the idea and enhanced the manuscript for submission. SQ was responsible for funding acquisition. All authors contributed to the article and approved the submitted version.
